The article "Study on the Application Value of PBL Combined with Situational Simulation Teaching Method in Clinical Practice Teaching of Radiology Department" was retracted in 2023. Reasons: unreliable results or conclusions; lack of ethics approval or compliance; concerns about the data; concerns about the peer review.

# Study on the Application Value of PBL Combined with Situational Simulation Teaching Method in Clinical Practice Teaching of Radiology Department

**DOI:** 10.1155/2022/6808648

**Published:** 2022-08-11

**Authors:** Tong Gong, Yuting Wang, Hong Pu, Longlin Yin, Mi Zhou

**Affiliations:** Radiology, Sichuan Provincial People's Hospital, University of Electronic Science and Technology of China, Chengdu 610072, China

## Abstract

**Objective:**

To study the application value of PBL (Problem-Based Learning) combined with a situational simulation teaching method in clinical practice teaching of radiology.

**Methods:**

120 interns who practiced in the radiology department of our hospital from 2020 to 2021 were randomly divided into a study group and a control group. The research group used PBL combined with the scenario simulation teaching method to carry out clinical practice teaching activities. The control group was carried out according to the conventional teaching plan. After 3 months, the teaching effect and satisfaction of the two groups were compared.

**Results:**

The imaging report quality control score, intravenous contrast agent score, and practice test score in the study group were higher than those in the control group. The scores of the small class and special class in the research group were higher than those in the control group, and the difference was statistically significant (*P* < 0.05). The scores of job competency questionnaire in the research group were higher than those in the control group (*P* < 0.05). The occupational self-efficacy questionnaire score of the research group was higher than that of the control group (*P* < 0.05). The nursing practice satisfaction score of the research group was higher than that of the control group (*P* < 0.05).

**Conclusion:**

The value of PBL combined with the scenario simulation teaching method in the teaching of radiology clinical practice is significant, which can improve the work ability of interns and make them more satisfied.

## 1. Introduction

With the continuous development of technology, radiological imaging examination has become an important auxiliary means in clinical diagnosis and treatment. Medicine has a stronger demand for postcompetency, and good postcompetence is the premise of providing quality medical services [1–3]. However, the imbalance of regional development will lead to the uneven ability of imaging graduates at the beginning of their clinical posts in radiology. With the continuous expansion of the enrolment scale of medical colleges and universities, improving the quality of practice has become one of the hotspots of medical education research [4–6].

The so-called internship refers to learning in the field or in practice [7, 8]. Internship can apply theoretical knowledge to work, which not only helps to deepen and consolidate book knowledge but also improves students' practical working ability to solve problems. Zhou believed that clinical practice meant that medical students completed the study of basic medical theory and entered the hospital to directly participate in the process of examination, diagnosis, and treatment of patients. In this process, medical students are required to have solid basic theoretical knowledge. They are also required to master the skills of examination, diagnosis, and treatment of patients [9]. With the development of clinical medicine and imaging examination technology, clinical imaging examination methods have been applied to a certain extent, which has greatly improved the diagnostic accuracy of the disease and been conducive to the early diagnosis of the disease. It has put forward new requirements for the training of radiology talents and promotes the implementation of the reform of medical education and teaching in radiology. With clinical practice as an important part of medical higher education, the quality of practice teaching is directly related to whether clinical interns can lay a solid foundation for practical medicine and determines the quality of medical college graduates [10]. Various problems have led to the poor quality of practice and low clinical skills of current imaging medical students [11–14]. Improving the quality of clinical teaching and practice in radiology has therefore become an urgent issue for medical educators to face and address.

PBL (Problem-Based Learning) is a problem-oriented way of learning. The most important feature of this teaching method is that it changes the passive learning of trainee students in the traditional teaching mode into active learning [15]. It has the advantage of exercising learning ability, communication skills, and teamwork ability [16]. Situational mimicry refers to the creation of situations similar to real-life scenarios in which students play various roles. This teaching mode will encourage students to actively explore and thus improve their ability to analyze problems independently, deal with problems, and communicate with each other [17]. In teaching practice, PBL teaching focuses on students' theoretical discussion and the content design of practical operation is a little weak, while situational simulation teaching focuses on students' practical training and is not enough for theoretical discussion. The Department of Radiology requires not only the superb professional level of medical staff but also its strong communication ability. It is more necessary to choose effective teaching methods to teach the trainee students in a relatively short time. The trained students achieve the general level of competence and operational skills required for clinical work. Therefore, this paper investigated the value of PBL combined with the situational simulation teaching method in the clinical practice teaching of radiology.

## 2. Materials and Methods

### 2.1. General Information

120 interns who practiced in the Department of Radiology in the hospital from 2020 to 2021 were randomly divided into a research group (*n* = 60) and control group (*n* = 60). There were 38 males and 22 females in the research group. In the control group, there were 40 males and 20 females. Inclusion criteria were as follows: (1) full-time imaging students, (2) students who can clearly express their true feelings, and (3) students who were able to understand and voluntarily participate in the entire process of this study and sign the informed consent form. Exclusion criteria were as follows: (1) the students who did not meet any of the inclusion criteria; (2) clinical practice nursing students who were unwilling to participate in this training due to personal reasons; (3) students who had ever PBL teaching and situational simulation teaching experience before; and (4) the students who were participating in other teaching and research. This study was a double-blind experiment.

### 2.2. Methods

#### 2.2.1. Technical Route

The technology roadmap is shown in Figure 1.

#### 2.2.2. Intervention Scheme

The interns of the control group received the traditional teaching mode after entering the department, including a small lecture once a week based on the teaching plan designated by each department. Special presentations were organized by the Department of Radiology.

PBL combined with the situational simulation teaching method was used to carry out clinical practice teaching activities in the research group. This teaching method can emphasize the student-centred approach. Clinical case group discussions and simulated clinical scenarios need to be integrated into the teaching process. The students can find answers through the analysis of cases and thus improve their own competence.

1. Preparation of intern students: (1) grouping: radiology interns were randomly assigned with about 9-11 students in each group; (2) PBL role assignment: this was determined by lottery within the group including 2 roles. One chairperson was responsible for maintaining classroom order, assigning work to students, leading students to collect information, and finally summarizing the results of everyone's discussions and making a report. One secretary was responsible for recording the ideas and opinions put forward by all students and removing roughness and extracting essence, the fake, and keeping the real work. All students participated in the discussion together and take turns to speak. (3) Situational simulation role assignment: the intern students were randomly divided into two groups. Each group takes turns explaining two scenarios, taking turns playing the roles of a doctor, patients, and family member
2. Teaching content arrangement: the classes were organized once a week, on Wednesday afternoon from 15:30 to 17:00. A total of five classes included one technical class and four theory classes. The radiology ward displays the classroom as a teaching venue
3. Teaching content: the imaging diagnosis of common diseases of single disease system was read, and 8 to 10 cases were selected each time according to cranial neoplastic lesions, cranial nonneoplastic lesions, head and neck lesions, pulmonary neoplastic lesions, pulmonary nonneoplastic lesions, hepatobiliary-pancreatic-splenic lesions, gastrointestinal lesions, genitourinary lesions, and common lesions of extremities/bone and joint. The format of the reading was verbal dictation. The dictation of the report simulated the process of writing a clinical report, describing both the signs and symptoms of the lesion and the diagnosis and differentiation of the disease. The clinical instructor conducted the film review. The work was divided and arranged for familiarity with imaging techniques, interpretation of signs and symptoms, standard use of imaging terminology, common diseases, diagnosis, and differential diagnosis of different diseases and adverse reactions to contrast media. The supervisor was expected to guide the trainee's thinking and to ask questions during the group review. The intern's mistakes were needed to be corrected at any time, and the relevant knowledge was explained briefly. Brainstorming was used to encourage students to put forward as many ideas and questions as possible; then, question them one by one and discuss them in the group at the same time. The secretary recorded the feedback. These questions were then further discussed and solved. After extensive data collection and information gathering, a summary was made to find out the most appropriate treatment method. The training of contrast application was divided into two stages, including theoretical teaching and first-aid exercises for adverse reactions to contrast agents. The theoretical training was first completed, followed by participation in the first aid exercise. According to the characteristics of the case and the development of the disease, a scenario simulation script was written and the characters were set according to the needs of the plot development. After the script was finalized, the teacher guided the students to memorize and recite the lines. When avoiding the performance, the students' performance was too exaggerated and false and the traces of the performance were too heavy, so that all the students' legal power was focused on the performance itself, while ignoring the solution of the problem. The training was organized twice a month. The performance of the residents participating in the exercise was rated according to the National Residency Clinical Competence (Intravenous Application of Contrast Media) scale

### 2.3. Observation Index

The main results are as follows: (1) quality control scores for the study image report, scores for the intravenous contrast agent, and scores for the practical examinations. All exams were scored on a percentage scale, except for the total score for intravenous contrast agents, which was 50 points. The internship examination results were composed of two parts, consisting of film reading assessment and theoretical assessment, each accounting for 50%. A total of 8 cases were examined, including 6 common diseases and 2 rare diseases with 10 points per question for common cases and 20 points per question for rare diseases. The types of imaging examination included X-ray, CT, and MRI. The types of questions in the theoretical examination included filling in blank questions, multiple choice questions, and short answer questions and examine the professional basis of imaging and the mastery of clinical application of physicians in resident Pei. The assessment used PPT reporting mode, and three senior attending physicians with professional titles or above were graded one by one according to the scoring criteria.

(2) The score of researches and special presentation. The highest scores of small and special presentation were 100, which were scored by three senior attending physician and above teachers according to the scoring criteria

(3) The score of “postcompetency questionnaire.” The postcompetency questionnaire included six evaluation items, such as operation ability, contingency ability, communication and coordination ability, management ability, job satisfaction, and scientific research ability [18]. The first five projects adopt the scoring model of 4 points (1-4 points) and whether the scientific research ability was evaluated. The higher the score, the stronger the competency of the position

(4) The score of professional self-efficacy questionnaire. The career self-efficacy questionnaire included 27 items in 6 dimensions, such as professional attitude and belief, problem-solving ability, career information collection and career planning ability, career cognition, career value, and career choice [19]. The score ranged from 27 to 135. Students with higher scores had stronger career self-efficacy

(5) The satisfaction score of nursing practice. Medical staff satisfaction scale was used to score, including work itself, work stress, interpersonal relationship, working conditions, work return, and organizational management [20]. There are a total of 6 evaluation dimensions and 20 closed items. The scale was scored by Likert five-level score (1~5 points). The higher the score, the better the satisfaction

### 2.4. Statistical Analysis

SPSS23.0 statistical software was adopted to process the data. The measurement data were presented as $\bar{x}\pm s$. The group design *t*-test was adopted for the comparison, and the analysis of variance was adopted for the comparison between multiple groups. The Dunnett test was adopted for comparison with the control group. The counting data were presented in the number of cases and the percentage, the *χ*^2^ test was adopted for comparison between groups, and bilateral test was employed for all statistical tests.

## 3. Results

### 3.1. The Quality Control Score of Image Report, the Score of Intravenous Application of Contrast Medium, and the Score of Practice Examination

After 3-month practice teaching, the quality control score of image report, the score of intravenous contrast medium, and the score of practice examination in the research group were significantly higher than those in the control group (*P* < 0.05, Table 1).

### 3.2. The Scores of Small and Special Presentations

After 3-month practice teaching, the scores of small and special presentations in the research group were obviously higher than those in the control group (*P* < 0.05, Tables 2–4).

### 3.3. The Score of the “Postcompetency Questionnaire”

Before practice teaching, there was no significant difference in the score of postcompetency questionnaire between the two groups (*P* > 0.05). After 3-month practice teaching, the score of the postcompetency questionnaire in the study group was remarkably higher than that in the control group (*P* < 0.05, Table 3).

### 3.4. The Score of the Career Self-Efficacy Questionnaire

There was no significant difference in the scores of the occupational self-efficacy questionnaire between the two groups before internship (*P* > 0.05). After 3 months of practice teaching, the score of the occupational self-efficacy questionnaire in the research group was considerably higher than that in the control group (*P* < 0.05, Table 4).

### 3.5. The Satisfaction Score of Nursing Practice

After 3 months of practice teaching, the satisfaction score of nursing practice in the research group was obviously higher than that in the control group (*P* < 0.05, Table 5).

## 4. Discussion

Radiology department is a department that integrates examination, diagnosis, and treatment [21]. Many diseases in clinical departments need to be diagnosed and assisted by radiological equipment [22–29]. With the aggravation of the medical tasks of the radiology department of the hospital, various examinations and evaluations are frequent. The clinical teaching time of the medical staff of the radiology department is not guaranteed, and the employment pressure leads to the “postgraduate entrance examination fever” and other factors, which consume most of the interns' time and energy, seriously affect the internship initiative, and then reduce the quality of internship [30, 31]. Clinical competence is a comprehensive ability that must be possessed in a series of special activities such as observation, understanding, judgment, and corresponding treatment of human health and diseases [32]. According to the American Board of Medical Examiners, medical students should have the following clinical competencies, including the ability to collect a medical history, physical examination, use of diagnostic ancillary tests, diagnostic skills, ability to make medical decisions, ability to implement medical decisions, ability to continue medical decisions, ability to continue treatment and care, proper management of the doctor-patient relationship, and professional attitude, the quality of which is reflected in clinical practice [33].

At present, the more traditional clinical practice teaching methods have been increasingly unable to meet the needs of nursing staff training required by the modern clinical practice of the Department of Radiology [34]. Although the traditional clinical practice teaching method is conducive to interns' rapid understanding and mastery of imaging diagnosis of common diseases of various systems, it tends to cause interns to develop habitual thinking and form the diagnostic mode of “looking at pictures.” This is not conducive to the cultivation of doctors' clinical imaging diagnostic thinking. There is also a lot of debate in academic circles about how to improve this traditional teaching model. Many educators and teaching researchers are trying to find better teaching methods to replace or improve the traditional teaching model [35]. Among them, PBL teaching method and situational simulation teaching method are more studied. In the late 1960s, Bruce put forward a new teaching method based on previous studies through many teaching practices, which emphasized that in the process of teaching, the students first need to be clear about the problem they are facing, and then, the teacher will freely divide the students into groups. The students study independently, and the whole teaching process is guided by teachers, namely, PBL teaching method. From the teaching level, the situational simulation teaching method means that in order to stimulate students' interest, teachers should provide students with a scientifically designed simulation situation, so that students can really feel in the situation, so as to achieve the goal of increasing students' knowledge and ability. These two methods improve students' comprehensive quality and thinking ability by stimulating their curiosity, interest in learning, and spirit of exploration. Therefore, combined with the clinical practice of radiology, this study creatively proposes the application of PBL teaching and situational simulation teaching to carry out clinical practice teaching in radiology clinical nursing teaching, providing a new method for clinical practice teaching in radiology. The results of this study showed that after the application of PBL teaching and situational simulation teaching, the interns' scores of image report quality, intravenous application of contrast medium, and practice examination were all higher than those of conventional clinical practice teaching. The scores of small and special presentations were higher than those of routine clinical practice teaching. The score of the “postcompetency questionnaire” was higher than that of routine clinical practice teaching, and the score of the occupational self-efficacy questionnaire was higher than that of routine clinical practice teaching. The satisfaction score of nursing practice was higher than that of routine clinical practice teaching. It is proven that the application value of PBL combined with situational simulation teaching method in radiology clinical practice teaching is significant. It is more helpful for interns to master image report quality, intravenous contrast agent application theory, and operation skills, improve clinical ability and teaching ability, improve interns' job competence, and improve interns' professional self-efficacy. In addition, it can make interns more satisfied with their internship work. This is mainly because traditional teaching focuses on mechanical repetition. The interns are easy to lose interest in learning, while PBL teaching method emphasizes that students play a leading role in the learning process by optimizing teaching links. Students discuss the clinical manifestations of the case in groups and summarize the imaging reading skills and points of attention for the use of contrast agents in the case. At the same time, the scenario simulation teaching method allows students to experience the feelings of different roles in the actual operation process, which is conducive to the improvement of students' learning motivation and the quality of teaching. Secondly, in the PBL joint scenario teaching process, students not only analyze clinical cases but also experience imaging techniques through scenario simulation. In the process of combining theory and practice, students can improve the application ability of imaging technology. Gao and other scholars have also reached the same conclusion as this study [21–23]. The study suggested that the test group's test scores after PBL teaching and scenario simulation teaching were significantly better than those of the control group. The study also mentioned that the application of PBL combined with scenario simulation teaching not only enhances students' understanding and application of theoretical knowledge but also rapidly improves students' practical skills. Thirdly, the PBL-combined scenario simulation teaching method can guide students to conduct independent learning by allowing students to consult literature, summarize data, and reproduce scenarios, thereby stimulating interns to analyze, explore, and create independently [25]. At the same time, the PBL-combined scenario simulation teaching method can more effectively stimulate students' curiosity and desire to explore. The students are more willing to take the initiative to analyze cases and check data by themselves in the scenarios they simulate to greatly improve their autonomous learning ability. The teaching quality and teaching efficiency of clinical practice can be improved, so that the interns are more satisfied with the practice work. This study still has some shortcomings. Firstly, the quality of this study is limited due to the small sample size we included in the study. Secondly, this research is a single-centre study, and our findings are subject to some degree of bias. Therefore, our results may differ from those of large-scale multicentre studies from other academic institutes. This research is still clinically significant, and further in-depth investigations will be carried out in the future.

To sum up, the value of PBL combined with the situational simulation teaching method in clinical practice teaching of radiology is significant. It is more conducive to the interns' mastery of the theoretical and operational skills of image report quality control, intravenous contrast application, improving the interns' working ability, and making them more satisfied with their internship.

## Figures and Tables

**Figure 1:** Technology roadmap.

**Table 1:** The quality control score of image report, the score of intravenous application of contrast medium, and the score of practice examination.

Grouping	Image report quality control score (points)	Intravenous contrast media score (score)	Internship examination results (points)
Control group (*n* = 60)	86.39 ± 2.17	40.15 ± 0.27	88.47 ± 1.44
Research group (*n* = 60)	93.42 ± 4.28	46.49 ± 1.65	96.53 ± 2.37
*χ* ^2^	11.348	29.373	22.513
*P* value	<0.01	<0.01	<0.01

**Table 2:** The scores of small and special presentations.

Grouping	Small presentation score (points)	Score of special presentation (points)
Control group (*n* = 60)	81.46 ± 2.27	82.43 ± 2.29
Research group (*n* = 60)	92.22 ± 3.17	90.39 ± 4.32
*t*	21.377	12.610
*P* value	<0.01	<0.01

**Table 3:** The score of the “job competency questionnaire”.

Grouping	Before internship and teaching	After 3 months of internship and teaching	*t*	*P* value
Control group (*n* = 60)	12.25 ± 0.19	18.68 ± 1.24	39.703	<0.01
Research group (*n* = 60)	12.28 ± 0.17	21.75 ± 2.04	35.834	<0.01
*t*	0.911	9.961		
*P* value	0.364	<0.01		

**Table 4:** The score of the career self-efficacy questionnaire.

Grouping	Before internship and teaching	After 3 months of internship and teaching	*t*	*P* value
Control group (*n* = 60)	70.52 ± 5.17	88.18 ± 6.23	16.897	<0.01
Research group (*n* = 60)	70.48 ± 5.22	108.46 ± 8.77	28.826	<0.01
*t*	0.042	14.603		
*P* value	0.966	<0.01		

**Table 5:** The satisfaction score of nursing practice.

Grouping	After 3 months of internship and teaching
Control group (*n* = 60)	72.46 ± 2.17
Research group (*n* = 60)	94.39 ± 3.99
*t*	37.400
*P* value	<0.01

## Data Availability

No data were used to support this study.
